This article has been retracted.

# Value of Neutrophil to Lymphocyte Ratio, Platelet to Lymphocyte Ratio, and Red Blood Cell Distribution Width in Evaluating the Prognosis of Children with Severe Pneumonia

**DOI:** 10.1155/2021/1818469

**Published:** 2021-09-24

**Authors:** Xuejiao Qi, Yihui Dong, Xiaojie Lin, Wencheng Xin

**Affiliations:** ^1^Department of Paediatrics, The Eighth People's Hospital of Qingdao City, Qingdao 266100, Shandong, China; ^2^Community Health Service Center of Qingdao Licang District, Yongqing Road, Qingdao 266041, Shandong, China

## Abstract

**Objective:**

To investigate the value of neutrophil to lymphocyte ratio (NLR), platelet to lymphocyte ratio (PLR), and red blood cell distribution width (RDW) in evaluating the prognosis of children with severe pneumonia (SP).

**Methods:**

A retrospective analysis of the data of 91 children with SP admitted to our hospital from March 2018 to March 2021. According to the survival status after 28 days of treatment, all children were divided into the survival group (*n* = 59) and the death group (*n* = 32). The clinical data and laboratory indicators of the patients were recorded. Multivariate logistic regression was used to analyze the risk factors of prognosis, and the ROC curve was used to analyze the predictive value of each index.

**Results:**

The Acute Physiology and Chronic Health Evaluation II (APACHE II) score and CURB-65 score of the death group were higher than those of the survival group (*P* < 0.05). The RDW, NLR, PLR, and high-sensitivity C-reactive protein, procalcitonin blood lactic acid (Lac) of the death group, were higher than those of the survival group, and LYM was lower than the survival group (*P* < 0.05). Multivariate regression analysis showed that APACHE II score, RDW, NLR, PLR, and Lac were all independent risk factors for poor prognosis in children with SP (*P* < 0.05). The AUC of NLR, PLR, and RDW for evaluating the prognosis of children with SP were 0.798, 0.781, and 0.777, respectively. The sensitivity was 56.25%, 90.63%, and 56.25%, respectively, and the specificity was 89.83%, 55.93%, and 91.53%, respectively. The AUC of NLR, PLR, and RDW combined to evaluate the prognosis of children with SP was 0.943. When the best cut-off value was 0.8528, the sensitivity was 93.75%, and the specificity was 91.53%.

**Conclusion:**

NLR, PLR, and RDW have certain predictive value for the prognosis of children with SP; the combination of the three indicators has a higher value in evaluating the prognosis of children with SP, which can better guide the prognostic treatment.

## 1. Introduction

Pneumonia is an infectious disease of the respiratory system caused by different pathogens such as bacteria and viruses, which can be caused by different causes. Because patients with pneumonia usually lack typical clinical manifestations in the early stage, patients are prone to gradual exacerbation of the disease due to improper treatment of empirical antibiotics and other reasons and even develop to a certain stage of disease, resulting in severe pneumonia (SP) [1, 2]. SP has hypoxia and acidosis as the main symptoms, which can affect lung parenchyma and oxygenation and, in severe cases, can lead to respiratory failure and dysfunction of multiple organs and even be life-threatening [3]. Studies have shown that 30% of deaths in the world are caused by infectious diseases at present, among which SP ranks the first in the mortality rate of infectious diseases. The disease age of SP is U-shaped, and it mostly occurs in children under 5 years old and elderly people over 65 years old [4, 5]. SP is characterized by rapid onset, rapid progression, many complications, and high morbidity and mortality. Therefore, it is particularly important to determine the severity of SP patients' condition at an early stage and evaluate the prognosis in time, so as to formulate comprehensive and effective treatment plans to reduce the mortality of patients.

Neutrophil to lymphocyte ratio (NLR) is a blood routine index reflecting systemic inflammation. The neutrophil count (NEU) can reflect the inflammatory state of the body. The more severe the inflammatory reaction, the higher the NEU count will be. The lymphocyte count (LYM) reflects the stress state of the body. The more severe the stress response, the lower the LYM count will be. NLR is easy to operate, low cost, and objective and has played an important role in the prognostic evaluation of tumor, diabetes, cardiovascular diseases, and respiratory diseases [6]. Platelet to lymphocyte ratio (PLR) is a related marker that reflects changes in platelet (PLT) and LYM counts. It can evaluate the severity of infectious diseases, as well as reflect or assess the degree of thrombosis and inflammatory response in the body. The higher the PLR, the higher the activation degree of PLT, the higher the risk of local vascular thrombosis, and the more obvious the ischemic changes caused by PLR [7]. Red blood cell distribution width (RDW) is a parameter that reflects the degree of dispersion of red blood cell size. The greater the value, the greater the heterogeneity of red blood cells. RDW is often used in the differential diagnosis of anemia in clinical practice and the value of stroke, autoimmune diseases, septic shock, and other diseases has attracted wide attention from scholars at home and abroad [8].

However, studies on whether NLR, PLR, and RDW can be used to determine the prognosis of children with SP are relatively rare. Therefore, this study reviewed the clinical information of 91 children with SP and evaluated the predictive value of NLR, PLR, and RDW in the risk of 28-day death in children with SP.

## 2. Materials and Methods

### 2.1. Research Object

A retrospective analysis of the data of 91 children with SP admitted to The Eighth People's Hospital of Qingdao City from March 2018 to March 2021 was performed. Among them, males (*n* = 53) and females (*n* = 38) were with an average age of 6.18 ± 3.26 years. According to the survival status after 28 days of treatment, all children were divided into the survival group (*n* = 59) and the death group (*n* = 32).

#### 2.1.1. Diagnostic Criteria

One of the following was met: invasive mechanical ventilation and septic shock that required the use of vasopressors. Otherwise, three of the following were met: respiration rate ≥ 30 times/min; oxygenation index (OI) ≤ 250 mmHg; multiple lung lobes infiltration; unconsciousness; blood urea nitrogen ≥ 200 mg/L; white blood cell count (WBC) < 4 × 10^9^/L; PLT < 10 × 10^9^/L; core body temperature < 36°C; and hypotension requiring body fluid resuscitation.

#### 2.1.2. Inclusion Criteria

The diagnostic criteria of SP were met [9]. Hospitalization time  > 24 h; age  < 10 years; the medical history data were complete; out-of-hospital treatment had no effect or did not receive treatment before admission; patients with increased or decreased WBC; and PLT were not caused by drugs.

#### 2.1.3. Exclusion Criteria

Active pulmonary tuberculosis; noninfectious interstitial pulmonary disease; pulmonary embolism; severe blood system disease; malignant tumor; use of immunosuppressive drugs; and had been treated in another hospital.

#### 2.1.4. Ethics

This study retrospectively analyzed the clinical data of the study subjects; without intervention on the children, informed consent could be exempted and approved by the ethics committee.

### 2.2. Research Methods

The clinical data of all children were obtained from the electronic medical record system of the hospital, and the gender, age, hospitalization days, and basic diseases of all children were recorded. The Acute Physiology and Chronic Health Evaluation II (APACHE II) score, Murray Lung Injury score, Sequential Organ Failure Assessment (SOFA), and CURB-65 score of all children within 24 hours of admission were recorded.

Laboratory indicators of the patient were recorded for 24 hours after admission: ① blood routine indexes: WBC, NEU, granulocyte ratio (GR%), LYM, PLT, RDW, NLR, and PLR were calculated, NLR = NEU/LYM and PLR = PLT/LYM; ② inflammatory indexes: high-sensitivity C-reactive protein (hs-CRP) and procalcitonin (PCT); ③ blood gas analysis indexes: blood lactic acid (Lac), OI was calculated, and OI = arterial oxygen tension (PaO_2_)/fraction of inspired O_2_ (FiO_2_).

### 2.3. Statistical Methods

SPSS22.0 software was used for analysis, measurement data were expressed as mean ± standard deviation, and *t* test was used for comparison. Count data were expressed as a ratio; *χ*^2^ test was used for comparison. Multivariate logistic regression was used to analyze the risk factors of prognosis, and the ROC curve was used to analyze the predictive value of each index. *P* < 0.05 was statistically significant.

## 3. Results

### 3.1. Comparison of Clinical Data between the Two Groups

There were no significant differences in gender, age, hospitalization days, and basic diseases between the two groups (*P* > 0.05), as illustrated in Table 1.

### 3.2. Comparison of Clinical Scores between the Two Groups

The APACHE II score and CURB-65 score of the death group were higher than those of the survival group (*P* < 0.05), as illustrated in Figure 1.

### 3.3. Comparison of Blood Routine Indexes between the Two Groups

The RDW, NLR, and PLR of the death group were higher than those of the survival group, and LYM was lower than the survival group (*P* < 0.05), as illustrated in Figure 2.

### 3.4. Comparison of Inflammatory Indexes between the Two Groups

The hs-CRP and PCT of the death group were higher than those of the survival group (*P* < 0.05), as illustrated in Figure 3.

### 3.5. Comparison of Blood Gas Analysis Indexes between the Two Groups

The Lac in the death group was higher than that in the survival group (*P* < 0.05), as illustrated in Figure 4.

### 3.6. Multivariate Analysis of Prognostic Factors in Patients with SP

Multivariate regression analysis showed that APACHE II score, RDW, NLR, PLR, and Lac were all independent risk factors for poor prognosis in children with SP (*P* < 0.05), as illustrated in Table 2.

### 3.7. Prognostic Value of Each Index in Patients with SP

The AUC of NLR, PLR, and RDW for evaluating the prognosis of children with SP were 0.798, 0.781, and 0.777, respectively. The sensitivity was 56.25%, 90.63%, and 56.25%, respectively, and the specificity was 89.83%, 55.93%, and 91.53%, respectively. The AUC of NLR, PLR, and RDW combined to evaluate the prognosis of children with SP was 0.943. When the best cut-off value was 0.8528, the sensitivity was 93.75%, and the specificity was 91.53%, as illustrated in Table 3 and Figure 5.

## 4. Discussion

With the change of lifestyle, SP has become a common clinical disease, which can not only cause damage to the respiratory system but also cause dysfunction of the nervous system and circulatory system. The mortality rate of SP ranks first among all types of pneumonia, and the prevalence has been increasing year by year in recent years, posing a serious threat to people's life and health [10, 11]. Even if the current medical technology continues to improve and the clinical treatment level of SP continues to increase, the morbidity and mortality remain high. Therefore, it is very important to diagnose and evaluate the prognosis of children with SP. Physicians in our department have rich experience in the field of critical diseases. This study evaluates the predictive value of different indicators for the prognosis of children with SP in order to provide a certain reference for clinical treatment.

In this study, APACHE II score, CURB-65 score, hs-CRP, PCT, Lac, LYM, and other indicators could be used to predict the prognosis of children with SP, but the above indicators had some limitations. The content of the APACHE II scoring system is complex, which is not conducive to rapid and simple assessment of disease condition and prognosis. Although the content of the CURB-65 scoring system is relatively simple, it is more suitable for outpatient applications. It can be used to assess whether patients need hospitalization, but may underestimate the risk of patients with basic diseases. As the precursor protein of calcitonin, PCT can reflect the infection situation of the body, with high sensitivity and specificity, but it is expensive, and the limited detection technology conditions lead to reduced scope of application, and it is not suitable for primary hospitals. hs-CRP, Lac, and LYM have low sensitivity or specificity and are affected by cost-effectiveness, clinical accessibility, and other factors, so they are not ideal indicators for the specificity evaluation of SP. Therefore, it is of great significance to find simple and feasible clinical markers to evaluate the prognosis of children with SP.

In the body of critically ill patients, a variety of factors will continuously induce the aggravation of the systemic inflammatory response, which will destroy the balance of defense immunity and regulation immunity, since NEU, LYM, and PLT play an important role in the regulation of inflammatory response, thus affecting the occurrence, development, and outcome of severe diseases. NEU and LYM are white blood cells in peripheral blood. NEU is mainly involved in innate immunity, that is, nonspecific inflammation reaction. Inhibiting NEU apoptosis and increasing NEU mediated killing are part of the innate immune response. LYM is an important cell in the human immune response and participates in adaptive immunity. When the body suffers from severe immune dysfunction and immunosuppression, it will trigger a series of pathological and physiological changes [12]. PLT occupies a central position in the initial stage and regulation of body inflammation and immune response. After pathogens are detected, PLT will be quickly activated and begin to drive the inflammatory response, directly regulating the activities of NEU, LYM, and endothelial cells ability, promoting the aggregation of a variety of adhesion molecules and chemokines to tissue damage and infection sites [13]. It is generally believed that NEU, LYM, and PLT are objective indicators reflecting the inflammatory response and immune state of the body in clinical practice. However, single detection indicators are easily affected by many factors, and the detection results have a large fluctuation range and low stability and are greatly affected by physiology and stress. Compared with NEU, LYM, and PLT, as ratio indicators, NLR and PLR can stably reflect the relationship between multiple factors and inflammatory response and immune system in the body. NLR is a combination of NEU and LYM; it can comprehensively express the balanced relationship between NEU and LYM and can quickly reflect the degree of inflammatory cell activation in patients, assess the severity of infectious diseases, and play a positive role in judging the prognosis of patients [14]. The increase of NLR often indicates the upregulation of NEU in the patient's body and the enhancement of the intensity of action, which has the characteristics of convenient acquisition and low cost, simple and fast [15]. The meta-analysis by Huang et al. [16] showed that for patients with sepsis, NLR may be an effective biomarker for prognostic evaluation, and the higher the value of NLR, the worse the prognosis of patients. When patients have an inflammatory disease, the peripheral blood circulation in the body is manifested as increased NEU and decreased LYM. Infection can lead to increased cytokine production and stimulate bone marrow megakaryocytes to produce PLT, and hypoxia can activate alveolar macrophages and release PLT activating factor; the basic protein kinase C activity of each component of PLT increases, so that PLT is activated, and the PLR value increases [17]. Smith et al. [18] first discovered in 2008 that preoperative PLR as an auxiliary indicator of tumor aggressiveness can improve the predictive value of serum CA19-9 in the laparoscopic examination of patients with potentially resectable periampullary malignancies. Kartal et al. [19] investigated 114 CAP patients and 50 healthy control subjects and found that the levels of NLR and PLR in CAP patients were significantly higher than those in the control patients, and there was a positive correlation between PLR and CRP. NLR and PLR could be used as predictors of CAP to predict the severity and prognosis of CAP. In addition, RDW is a parameter to measure the volume heterogeneity of red blood cells in a short period of time using a blood cell counter. The larger the RDW, the greater the volume variability of red blood cells will be. RDW can affect the level of inflammatory factors in the body, which is very important for the prognosis of infectious diseases. When the patient is infected, the blood system is abnormal, the environment of red blood cells is changed, the number of red blood cells is reduced, and the compensation causes an increase in small red blood cells, which reduces the plasticity of red blood cells, leading to the increase of RDW [20]. RDW can be obtained by blood routine test results, without additional testing costs. It has the characteristics of simplicity, convenience, low cost, and easy testing and has been widely used in the diagnosis and prognosis prediction of cardiopulmonary diseases and peripheral vascular diseases. Zhang et al. [21] found that the RDW of patients who died of severe acute pancreatitis was higher than that in patients who survived; there was a significant relationship between RDW and APACHE II and SOFA scores, which had good prognostic value. Since most of the SP patients are accompanied by basic diseases, in order to eliminate the influence of these factors, this study balances the proportion of the basic diseases of the two groups of SP children, so as to eliminate their interference to the results to the maximum extent. In this study, the RDW, NLR, and PLR of the death group were higher than those of the survival group, and RDW, NLR, and PLR were all independent risk factors for poor prognosis in children with SP. The results showed that RDW, NLR, and PLR are closely related to the prognosis of children with SP. However, due to the short half-life of PLT, the number of PLT is affected by a variety of factors, such as bacterial endotoxins and inflammatory reaction, which can lead to the decrease of the number of PLT. Therefore, the value of PLR varies greatly, and its diagnostic efficacy as an indicator of inflammation may be lower than that of NLR, and further verification is still needed.

Studies have shown [22] that the AUC values of NLR, PLR, and RDW for predicting the 28-day mortality of patients with acute pancreatitis were 0.851, 0.693, and 0.885, respectively. However, the detection of clinical indicators alone has limited significance in predicting the prognosis of patients, and there are certain limitations in the diagnosis and treatment of the disease, and the combination of multiple indicators for prediction can significantly improve the evaluation value. The results of this study showed that the AUC of NLR, PLR, and RDW for evaluating the prognosis of children with SP were 0.798, 0.781, and 0.777, respectively, and the AUC of NLR, PLR, and RDW combined to evaluate the prognosis of children with SP was 0.943. We believe that NLR, PLR, and RDW have certain predictive value for the prognosis of children with SP. In this study, it was found that the combination of NLR and PLR combined with RDW has the largest AUC for the diagnosis of SP children, with an AUC of 0.943, and had good sensitivity and specificity. Compared with single indicator, the combination of three indicators has a higher value in evaluating the prognosis of children with SP. In clinical treatment of SP children, medical staff should pay close attention to the dynamic changes of these three indicators of NLR, PLR, and RDW. The measurement of these indicators is simple, cheap, economical, rapid, and easy to obtain, and they are relatively ideal markers in clinical use, which can better guide the prognostic treatment and implement a better intervention plan for children, so as to improve the outcome of children, and easy to promote in primary hospitals.

## 5. Conclusion

In summary, NLR, PLR, and RDW have certain predictive value for the prognosis of children with SP; the combination of three indicators has a higher value in evaluating the prognosis of children with SP, which can better guide the prognostic treatment. However, there are certain shortcomings in this study. The subjects of the study are limited to SP children in our hospital; the sample size is relatively small; it was a retrospective analysis, and many factors affecting the survival of SP children have not been comprehensively considered. Therefore, the results of this study still need to be verified by a larger prospective study and exclude other factors for a comprehensive discussion of the prognosis.

## Figures and Tables

**Figure 1:** Comparison of clinical scores between the two groups. Note: compared with the survival group, ^*∗*^*P* < 0.05.

**Figure 2:** Comparison of blood routine indexes between the two groups. Note: compared with the survival group, ^*∗*^*P* < 0.05.

**Figure 3:** Comparison of inflammatory indexes between the two groups. Note: compared with the survival group, ^*∗*^*P* < 0.05.

**Figure 4:** Comparison of blood gas analysis indexes between the two groups. Note: compared with the survival group, ^*∗*^*P* < 0.05.

**Figure 5:** Prognostic value of each index in patients with SP.

**Table 1:** Comparison of clinical data between the two groups (*n*, %, $\bar{x}\pm s$).

Clinical data	Survival group (*n* = 59)	Death group (*n* = 32)	*χ*^2^/*t* value	*P* value
Gender			0.368	0.544
Male	33 (55.93%)	20 (62.50%)		
Female	26 (44.07%)	12 (37.50%)		
Age (years)	6.70 ± 3.57	5.22 ± 3.14	1.967	0.052
Hospitalization (days)	13.02 ± 10.25	11.38 ± 9.14	0.756	0.451
Basic diseases			0.771	0.942
Hypertension	25 (42.37%)	14 (43.75%)		
Diabetes	13 (22.03%)	8 (25.0%)		
Cerebrovascular disease	9 (15.25%)	5 (15.63%)		
Chronic obstructive pulmonary disease	7 (11.86%)	2 (6.25%)		
Coronary heart disease	5 (8.47%)	3 (9.38%)		

**Table 2:** Multivariate analysis of prognostic factors in patients with SP.

Variable	*B* value	SE value	Walds value	OR value	95% CI	*P* value
APACHE II score	0.336	0.089	14.252	1.399	1.175∼1.666	0.009
CURB-65 score	0.248	0.133	3.476	1.281	0.987∼1.663	0.069
LYM	0.370	0.265	1.949	1.447	0.861∼2.434	0.073
RDW	0.294	0.118	6.207	1.342	1.064∼1.690	0.038
NLR	0.315	0.126	6.250	1.370	1.070∼1.754	0.021
PLR	0.302	0.134	5.079	1.352	1.040∼1.758	0.043
hs-CRP	0.381	0.217	3.082	1.463	0.956∼2.239	0.144
PCT	0.253	0.142	3.174	1.287	0.975∼1.701	0.163
Lac	0.199	0.101	3.882	1.220	1.001∼1.487	0.045

**Table 3:** Prognostic value of each index in patients with SP.

Index	AUC	Asymptotically 95% CI		Best cut-off value	Sensitivity (%)	Specificity (%)
		Lower limit	Upper limit			
NLR	0.798	0.699	0.896	0.4608	56.25	89.83
PLR	0.781	0.682	0.879	0.4656	90.63	55.93
RDW	0.777	0.673	0.882	0.4778	56.25	91.53
NLR + PLR + RDW	0.943	0.881	1.000	0.8528	93.75	91.53

## Data Availability

The data used and/or analyzed during the current study are available from all the authors.
